The article "Bioinformatic Analysis of PTTG Family and Prognosis and Immune Cell Infiltration in Gastric Cancer" was retracted in 2024. Reasons: signs of a paper mill; suspected computer-generated content; unreliable results or conclusions; concerns about the data.

# Bioinformatic Analysis of PTTG Family and Prognosis and Immune Cell Infiltration in Gastric Cancer

**DOI:** 10.1155/2023/6905216

**Published:** 2023-02-04

**Authors:** Xiao Li, Yanghao Tai, Shuying Liu, Yating Gao, Kaining Zhang, Jierong Yin, Huijuan Zhang, Xia Wang, Xiaofei Li, Dongfeng Zhang

**Affiliations:** ^1^Department of Thoracic Oncology, Linfen Central Hospital, Linfen 041000, China; ^2^Shanxi Medical University, Taiyuan 030000, China

## Abstract

Gastric cancer is the sixth highest incidence rate in the world. Although treatment has made progress, the prospect of gastric cancer patients is bleak. Difficulties and future prospects of immunotherapy in cancer treatment. Adaptive cell therapy, cancer vaccines, gene therapy, and monoclonal antibody therapy have all been used in gastric cancer with some initial success. PTTGs (pituitary tumor-transforming genes) have been proven to be closely related to the prognosis of many malignant tumors. However, the prognosis and immune cell infiltration of gastric adenocarcinoma (STAD) remain unclear. We retrieved multiple databases to understand the possible activity of PTTGs and their expression in gastric cancer, as well as their relationship with clinical data, overall survival rate, first progression, and survival rate after progression. PTTGs are overexpressed in STAD tumor tissues. Many clinical variables are closely related to PTTGs. In addition, PTTG was associated with overall survival independent of disease. In addition, the expression of PTTG1/2 was positively correlated with the molecular status of the immune checkpoint and negatively correlated with the infiltration of various immune cells. Data research shows that PTTG and STAD are closely related. This paved the way for future research, revealed the complex pathophysiology of gastric cancer, and introduced an effective new treatment.

## 1. Introduction

At present, according to the data released by the International Agency for Research on Cancer (IARC), more than 1,033,701 new cases of gastric cancer were reported in 2018, and about 800,000 people died of gastric cancer [1]. In 2018, about 10% of cancer deaths are caused by gastric cancer, which makes gastric cancer the sixth largest cancer in the world. After lung cancer and colorectal cancer, it is the third leading cause of cancer-related mortality [2]. Epidemiological studies show that in 2018, the incidence rate of gastric cancer was 11.1%/100,000 and the mortality rate was 8.2%/100,000. High incidence areas and mortality are mainly concentrated in East Asia, Eastern Europe, and South America. The proportion of men suffering from gastric cancer is twice that of women [2]. In terms of treatment, the effective rate and R0 resection rate of the FLOT regimen (5-fluorouracil, folic acid, oxaliplatin, and docetaxel) are higher than those of standard ECF and epirubicin, 5-fluorouracil, and capecitabine (ECX) [3]. Nevertheless, the prognosis of gastric cancer is still poor, with a median survival of about one year. Claudin ­ 18.2 (more common in diffuse cancer) is the inhibitor of fibroblast growth receptor 2 pathway, antiangiogenesis therapy, and immune checkpoint inhibitor, which is the key to the treatment of cancer [4–7].

There are now three genes known to make up the pituitary tumor-transforming gene (PTTG) family [8, 9]. These genes are pituitary tumor-transforming 1 (PTTG1), pituitary tumor-transforming 2 (PTTG2), and pituitary tumor-transforming 3P (PTTG3P). PTTG1 is homologous to PTTG2 and PTTG3P [9], and it has been shown to be upregulated in numerous endocrine-related malignancies in both domestic and international investigations. Little is known about the biological roles of PTTG2; however, it and its related protein, PTTG3P, have been linked to the emergence of many human cancers.

Current research shows that PTTG1 and PTTG2 participate in the carcinogenic process [10–12], and PTTG3P, as an intron-free gene with high homology between PTTG1 and PTTG2, also participates in some processes [13]. PTTGs are overexpressed in many cancers, such as lung cancer, gastric cancer, kidney cancer, pancreatic cancer, breast cancer, liver cancer, and esophageal cancer [14–18]. They are involved in all stages of cells. The imbalance of PTTG1 enhances the proliferation, invasion, and metastasis of tumor cells and inhibits apoptosis [19–21]. PTTG2 and PTTG3P are homologous genes of PTTG1 [8]. Although their functions are not well understood, they have been confirmed to be closely related to the development of human cancer. Guo et al. [12] proved that PTTG2 was significantly upregulated in glioblastoma, and its overexpression promoted the proliferation and invasion of glioblastoma cells. Weng et al. [14] proved that PTTG3P can enhance the proliferation and invasion of GC in vitro, which is an indicator of poor prognosis. Xu et al. [22] found that PTTG1 mRNA expression in four of the six human GC cell lines was significantly higher than that in their low count cells, consistent with the data of mRNA expression.

This article uses bioinformatic analysis to shed light on the connection between PTTGs and several aspects of gastric cancer, including gene expression, clinical data analysis, prognosis, immune infiltration, etc. This research shows that PTTGs significantly influenced the onset and progression of gastric cancer which opens up new avenues for research into stomach cancer, sheds light on its complex pathophysiology, and points toward potential therapeutic interventions.

## 2. Methodology

### 2.1. Oncomine Analysis

Oncomine (https://www.oncomine.org/) is an independent access microarray resource for tumor-associated gene expression profiles and linked clinical data. Tumor and normal tissue samples were analyzed using Oncomine to compare the PTTG family gene transcription. Changes in expression levels are considered statistically significant when the fold change is greater than 1.5 and the *p* value is less than 0.05. We set the gene level threshold to “top 10%” and the data type to “mRNA.”

### 2.2. GEPIA Analysis

GEPIA (Gene Expression Profiling Interactive Analysis) (http://gepia.cancer-pku.cn/index.html), which is based on the GTEx (Genotype-Tissue Expression) and TCGA (The Cancer Genome Atlas) datasets, was implemented to examine the correlation between the sequencing of PTTGs in gastric cancer (GC) tissues and individual tumor stages. GEPIA is implemented to compare the expression level of PTTGs in gastric cancer tissues and normal tissues with the threshold of |log2(fold change)|. The critical value is 1 and the *p* value critical value is 0.01. The default parameters were used to analyze the expression of PTTGs in gastric cancer tissues and normal tissues.

### 2.3. UALCAN Database

Based on level 3 RNA sequences and clinical data for 31 malignancies included in the TCGA database, UALCAN (the University of Alabama at Birmingham Cancer data analysis portal) (http://ualcan.path.uab.edu) is an interactive online resource. Main applications include comparing gene expression levels in tumor and normal tissue samples and determining whether or not there is a relationship between gene expression and clinicopathological variables. In this investigation, we utilized UALCAN to examine the mRNA expressions of PTTG family members in STAD carcinoma tissues and the correlations between these expressions and the presence or absence of cancer in the lymph nodes. In the experiment conducted by the students, the *p* value threshold was established at 0.01.

### 2.4. Kaplan-Meier Plotter Analysis

We utilize the Kaplan-Meier plotter (http://kmplot.com/analysis/) to compare the predictive significance of various PTTG family gene expression levels across three time points: overall survival (OS), time to first progression (FP), and time to second progression (PPS). Group patients by automatically selecting the best cut-off value. The minimum required for further communication is all. Hazard ratio: Yes; 95% confidence interval: Yes. Available probe sets include only the highest-quality JetSet brand probes.

### 2.5. cBioPortal Analysis

The TCGA database's biomolecules in tumor tissues may be analyzed interactively using cBioPortal (http://www.cbioportal.org/). Here, we use it to analyze the changes in the frequency of PTTG gene changes. We compared the impact of altering the default settings on STAD patients' prognosis and survival in the comparison/survival module.

### 2.6. TIMER 2.0 Analysis

We used TIMER 2.0 (Tumor IMmune Estimation Resource) (http://timer.comp-genomics.org/) to examine the correlation between PTTG expression in STAD tissues and the number of immune cells present. Analysis of biomarker gene expression in the TIMER database is utilized to calculate the extent of tumor invasion. Here, we use the immunological correlation module to look for cancer cells by selecting PTTG1, PTTG2, or PTTG3P as the input. In this experiment, we chose to use B cells, CD8+ T cells, CD4+ T cells, neutrophils, macrophages, and dendritic cells. The log2 TPM value is derived from the expression level of the genes in question. Finally, we analyzed the relationship between the expression of PTTGs and the expression of specific markers of immune infiltrating cell subsets.

### 2.7. GeneMANIA Analysis

To find genomic correlations and look for similarly expressed proteins, researchers utilize GeneMANIA (http://genemania.org/), which is built on a plethora of huge publicly accessible biological datasets. Here, we utilize GeneMANIA with its default settings to find PTTGs that interact with one another and are coexpressed in the human dataset.

### 2.8. STRING

The dataset of the Search Tool for the Retrieval of Interacting Genes/Proteins (STRING, https://string-db.org/), an interactive online server, is suitable for visualizing, exploring, and analyzing the interaction between various proteins and equivalent genes. We likewise utilized STRING to design a protein-protein interaction network including the two seed genes (PTTG1 and PTTG2) and their top 10 functional partners according to their levels of confidence (scoring > 0.900). Insightful information on STAD's development may be gleaned from the interconnectedness of PTTG and neighboring genes. This PTTG-neighbor gene network model is built using the STRING website with the following parameters: the minimum required interaction score is 0.900; the maximum number of interactors to be displayed is the second shell-none; the meaning of network edges is evidence; active interaction sources are text mining, experiments, databases, coexpression, neighborhood, cooccurrence, and gene fusion; and the minimum required interaction score is 0.900.

### 2.9. DAVID

From the cBioPortal database, we selected the top 50 genes linked to PTTGs. Using the DAVID database (https://david.ncifcrf.gov/summary.jsp), the functions of PTTGs and 50 related proteins were examined using Gene Ontology (GO) and Kyoto Encyclopedia of Genes and Genomes (KEGG). Biological process (BP), cellular component (CC), and molecular function (MF) enrichment analyses could predict the function of PTTGs and their 50 linked proteins, while KEGG analysis could reveal the connected pathways of PTTGs and their associated interactors.

## 3. Results and Discussion

### 3.1. Differential Expressions of PTTGs in GC

Figure 1 and Table 1 display the Oncomine database findings. We addressed the issue of multiple testing by using the FDR technique. PTTG1 mRNA expression was shown to be significantly greater in GC tissues across different datasets (Figure 1). The expression of PTTG1 in gastric mixed adenocarcinoma tissues was significantly higher than that in normal controls (2.0-fold, *p* = 6.17*E* − 07) in Chen's gastric dataset. Cho et al. also showed that PTTG1 is significantly increased in gastric mixed adenocarcinoma compared to normal controls (fold change = 2.064, *p* = 0.001). Diffuse gastric cancer is associated with an upregulation of PTTG1 (fold change = 2.367, *p* = 1.98*E* − 06), as reported by Cho et al. What is more, PTTG1 was overexpressed in gastric intestinal-type adenocarcinoma tissues than in the normal tissues in many datasets: by a fold change of 2.321 (*p* = 2.41*E* − 17) in the Chen gastric dataset [23], by a fold change of 1.790 (*p* = 0.002) in the Cho dataset [24], and by a fold change of 2.631 (*p* = 2.24*E* − 10) in the D'Errico dataset [25]. It was also shown that PTTG2 was significantly upregulated in GC tissues compared to normal tissues. In addition, both diffuse gastric adenocarcinoma and gastric intestinal-type adenocarcinoma showed an upregulation of PTTG3P (fold change = 2.323, *p* = 3.67*E* − 05, and fold change = 3.234, *p* = 3.39*E* − 07, respectively) (Table 1).

The GEPIA2 dataset results showed that PTTG1 mRNA levels were higher in STAD tissues compared to normal controls, whereas PTTG2/3P transcript levels were not different between STAD (stomach adenocarcinoma) tissues and normal tissues (Figure 2). Multiple testing was adjusted for using the FDR method.

### 3.2. Prognostic Value of mRNA Expression of PTTGs in STAD Patients

We aimed to clarify the connection between PTTG mRNA levels and STAD tumor progression.  Figure 3(a) demonstrates that, contrary to our expectations, we did not find any statistically significant correlations between PTTG mRNA levels and tumor stages (*p* > 0.01). Moreover, we discovered that improved OS, FP, and PPS (*p* < 0.05) were associated with elevated PTTG1 and PTTG3P transcription levels in GC patients (Figure 4), meanwhile elevated PTTG2 transcription levels were detrimental to GC patients' overall survival (OS), progression-free survival (PFS), and progression-to-stage (PPS) (*p* < 0.05) (Figure 4).

### 3.3. Correlation of PTTG Expression and Prognosis with Different Clinicopathological Factors in Gastric Cancer Patients

Using the TCGA database, we analyzed the correlation between PTTG expression and clinical features with the use of the Kaplan-Meier plotter to get a deeper understanding of the significance of complement expression in cancer. Improvements in OS were seen across gender, stage, stage T2/3, stage M, and Lauren categorization when the PTTG1/3 expression was elevated (*p* < 0.05). Also, higher PTTG1 expression was linked to longer OS in GC patients at stage N (Table 2, *p* < 0.05).  Figure 3 demonstrates that the expression of PTTGs is inversely related to the severity of STAD pathology. According to the patient's pathological status, this function may produce an expressive violin plot. The initial tumor's size or direct spread is what the T stage indicates here. High levels of PTTG2 expression are associated with worse OS across all genders, stages, and histologies but especially in stage 1/3 and N0. The improved OS N1/3/1 + 2 + 3 stage was due to increased expression of PTTG3P. Further, lymph node involvement is denoted by the N category; N0 shows that tumor cells are not present in regional lymph nodes, whereas N1 through N3 indicate that metastases have spread to regional lymph nodes.

### 3.4. Gene Mutation of PTTGs and Its Significance in the Prognosis of STAD Patients

We used the cBioPortal online tool for STAD (TCGA, Pan-Cancer Atlas; https://www.cbioportal.org) to evaluate PTTG gene alterations and their significance to OS and DFS. Out of a total of 412 individuals with STAD, 67 patients (16%) were determined to have a mutated gene (Figure 5(a)). The gene mutation rates of PTTG1, PTTG2, and PTTG3P were 6%, 5%, and 9%, respectively.  Figure 6(a) demonstrates that PTTG gene changes were most common in patients with diffuse-type stomach adenocarcinoma, occurring in 24.64% of 69 cases. The shortened DSS (Figure 5(f), *p* = 0.0108) but not the shortened OS (Figure 5(c), *p* = 0.100), DFS (Figure 5(d), *p* = 0.359), or PFS (Figure 5(e), *p* = 0.127) of STAD patients was linked with genetic abnormalities in PTTGs.

### 3.5. Correlation between PTTG Expression and Immune Infiltration in STAD

As immune cells are linked to tumor growth and spread, we used TIMER to examine the relationship between PTTG family members and immune infiltration in STAD. It came as a surprise to us that the amount of expression of the PTTG family had no effect on the degree of tumor purity. As can be seen in Figure 6(a), we found a negative correlation between PTTG1 expression and the percentage of B cells, CD4+ T cells, macrophages, and dendritic cells infiltrating STAD, but not with CD8+ T cells (Cor = −0.083, *p* = 1.11*E* − 01), and neutrophils (Cor = −0.059, *p* = 2.57*E* − 01). Not only was there a positive correlation between PTTG2 expression and the infiltration of CD8+ T cells (Cor = 0.173, *p* = 8.30*E* − 04), CD4+ T cells (Cor = 0.13, *p* = 1.27*E* − 02), macrophages (Cor = 0.264, *p* = 2.58*E* − 07), neutrophils (Cor = 0.198, *p* = 1.22*E* − 04), and dendritic cells (Cor = 0.207, *p* = 5.77*E* − 05) (Figure 6(b)), there was also a lower-than-average connection between PTTG3P expression with any of the six categories of immune cells (Figure 6(c)). Moreover, KM survival analysis reveals a significant correlation between the macrophage (log-rank *p* = 0.002) and dendritic cell (log-rank *p* = 0.022) infiltration and the prognosis of patients with gastric cancer (Figure 6(d)).

### 3.6. Examining the Association between mRNA Levels of PTTGs and Immune Cell Subset Markers

The TIMER database was queried to find more evidence linking PTTG expression with immune cell infiltration level, using the STAD collection of immunologic markers as a starting point. We looked examined how PTTG expression compared to other markers in several cell subsets, including CD8+ cells, T cells (general), B cells, monocytes, TAM, M1 macrophages, M2 macrophages, neutrophils, natural killer cells, and democratic cells. We looked at T helper 1 (Th1) and T helper 2 (Th2) cells, as well as follicular helper T (TFH) cells, T helper 17 (Th17) cells, regulatory T (Treg) cells, and T cell fatigue. Since the immune osmotic analysis is affected by the tumor purity of clinical samples, we accounted for this in our adjustments. According to the findings, most marker genes in immune osmotic cells were substantially correlated with the expression of PTTGs in STAD tissues (Table 3).

Most indicators for B cells, monocytes, M2 macrophages, and neutrophils were linked with PTTG1 expression in STAD (Table 2). In particular, it was highly linked with markers for B cells (CD879A), monocytes (CD115), and neutrophils (ITGAM, CCR7) in STAD (*p* < 0.0001). The expression of PTTG2 in STAD was also shown to be substantially linked with the expression of immunological marker genes in T cells, monocytes, M2 macrophages, neutrophils, natural killer cells, and dendritic cells. Specifically, the PTTG1 level in STAD was correlated with CD3D and CD2 of T cells; CD86 of monocytes; CD163 and MS4A4A of M2 macrophages; CEACAM8 of neutrophils; KIR2DL1, KIR2DL3, and KIR3DL2 of natural killer cells; and NRP1 of dendritic cells (*p* < 0.0001). To a large extent, natural killer cell immune markers are correlated with the PTTG3P expression. The correlation between KIR2DL1 and KIR2DL3 was very strong (*p* < 0.0001). The expression of PTTGs was significantly connected with the expression of Th1 markers (STAT1 and IFNG), Th2 markers (STAT6 and STAT5A), Tfh markers (BCL6 and STAT3), the Treg marker (STAT5B), and the T cell exhaustion marker (GZMB) (*p* < 0.0001). Unfortunately, we found that the expression of PTTG2 and PTTG3P had little significant correlation with T cell immune markers in different subsets.

### 3.7. Gene and Protein-Protein Interaction Network of PTTGs

As an added bonus, the gene–gene interaction network of PTTGs is obtained through GeneMANIA. The disadvantage is that PTTG3P is an unrecognized gene in the two databases. The physical relationships, coexpression, predictions, colocalization, route, genetic connections, and common protein domains between PTTGs and the 20 genes around them are shown in Figure 7(a) as 20 additional nodes. The five genes with the strongest associations with PTTGs were found to be ESPL1 (extra spindle pole bodies like 1), DECR1 (2,4-dienoyl-CoA reductase 1), CDC27 (cell division cycle 27), CDC20 (cell division cycle), and ZWINT (ZW10 interacting kinetochore protein), among which PTTG1 was linked with PTTG2 for pathway, physical interactions, and predictions. In addition, the results of the functional analysis revealed a significant relationship between these genes and nuclear ubiquitin ligase complex, mitotic sister chromatid separation, and chromosome separation.

We also performed a protein-protein interaction network using STRING between the seed genes (PTTG1 and PTTG2) and their top 10 functional partners with the highest confidence ratings (score > 0.900, Figure 7(b)). Extra spindle pole bodies like 1 (ESPL1), FZR1 (fizzy-related protein homolog), ANAPC11 (anaphase-promoting complex subunit 11), Aurora kinase A (AURKA), and ANAPC2 (anaphase-promoting complex subunit 2) were the top five proteins in terms of their strongest connections with the PTTGs (anaphase-promoting complex subunit 2). Based on the findings, the following biological processes were shown to be mostly dependent on the PPI network: anaphase-promoting complex-dependent catabolic process, nuclear division, cell cycle process, mitotic sister chromatid separation, and mitotic cell cycle, and the main KEGG pathways were ubiquitin-mediated proteolysis, oocyte meiosis, cell cycle, human T cell leukemia virus 1 infection, and progesterone-mediated oocyte maturation.

### 3.8. Examination of PTTGs and Related Genes in STAD Patients via Enrichment Analysis

Improved understanding of the biological functions of PTTGs may help to clarify their potential mechanisms in STAD. Subsequently, 50 coexpression genes of specific PTTG molecules in STAD were selected through the cBioPortal database. The DAVID database was applied for GO and KEGG enrichment analyses of PTTG family members and their relative genes (Figure 8). The results showed that PTTG molecules could affect the following processes in STAD.

These genes were shown to have crucial roles in biological processes such as cell division, mitotic nuclear division, and sister chromatid cohesion. Each of the cell's constituent parts—the nucleus, the cytoplasm, the cytosol, and the nucleoplasm—played a role in all of these. Binding proteins, poly(A), and adenosine triphosphate (ATP) were all molecular functions. Genes that were coexpressed by PTTG1/2/3P were found to be abundant in signalling pathways involved in cell cycle regulation, oocyte meiosis, progesterone-mediated oocyte maturation, and viral carcinogenesis, according to the KEGG analysis.

## 4. Conclusion

Using several databases, we compared PTTG expression in tumor and normal tissues and determined whether or not there was a link between PTTG mRNA expression and the tumor stage in STAD patients. The purpose of this study was to detect the relationship between the expression of PTTG family members and OS, FP, and PPS in patients with STAD, predict the relationship between PTTG expression and clinical prognosis of gastric cancer using several clinicopathological parameters, and detect the relationship between PTTG transcriptional expression and gene mutation frequency and the overall survival rate of patients with STAD. At the same time, we looked at how PTTGs might work, how they might be expressed, and how they might relate to markers on immune cells that are known to infiltrate tumors. It was discovered that STAD tumor tissues have higher levels of PTTG1/2/3P. A high expression of PTTG1/3P was linked to improved overall survival (OS), progression-free survival (PFS), and post-progression survival (PPS) in a survival analysis. The inverse is true when PTTG2 expression levels are elevated. Based on the analyzed clinical data, it was discovered that an increased expression of PTTG1/3 was related to a correlation between OS and gender, stage, T2/3, M, and Lauren grading, while an increased expression of PTTG2 was related to a correlation between OS and gender, 1/3, and N0, but had a weaker effect on OS. Furthermore, PTTG mutations were analyzed. The modified group had a lower disease-specific survival (DSS) rate than the control group. Gene Ontology and Kyoto Encyclopedia of Genes and Genomes analyses revealed that PTTGs participated in several different genetic pathways, such as the cell cycle, oocyte meiosis, and progesterone-mediated oocyte maturation. It was also found that the expression of immune checkpoints was positively correlated with the expression of PTTG1/2, while the expression of various immune cells that had antitumor effects was negatively correlated with the expression of PTTG1/2. We found that PTTGs significantly influenced the onset and progression of gastric cancer through our analysis of these genes. This opens up new avenues for research into stomach cancer, sheds light on its complex pathophysiology, and points toward potential therapeutic interventions.

## Figures and Tables

**Figure 1:** (a) The mRNA expression levels of PTTGs in 20 distinct cancer illnesses (Oncomine). The graph displays the number of datasets with elevated (red) and downregulated (blue) changes in the target gene's mRNA expression that is statistically significant. Student's *t*-test was used to compare variations in mRNA levels. The following settings were chosen: *p* < 0.05, fold change = 1.5, gene rank = 10%, and data type = mRNA. The false discovery rate (FDR) approach was used to perform the multiple testing adjustment. (b) PTTG1 mRNA expression in GC was meta-analyzed using data from various Oncomine databases.

**Figure 2:** Evaluation of PTTG mRNA expression in STAD tissues against normal stomach tissues (GEPIA2). The mRNA expression of PTTGs was compared in STAD tissues and healthy controls using a scatter diagram (a) and a box plot (b). The false discovery rate (FDR) technique was used to adjust for multiple testing. The following conditions were established: We found a significant correlation between the two sets of data (*p* = 0.01, |log2*FC*| = 1), indicating that normal data from TCGA and GTEx patients are similar. (b) Tumor tissues are shown in red, whereas normal tissues are shown in grey. There is statistically significant difference between (a) and (b), as shown by the pink STAD and ∗, respectively. T: tumor samples; N: normal samples; STAD: stomach adenocarcinoma; TPM: transcripts per million. (c) Comparison of PTTG expression between STAD and healthy tissues (UALCAN).

**Figure 3:** Clinicopathological characteristics associated with STAD and the expression of PTTGs. (a) The correlation of PTTG mRNA expression with tumor grade in individuals with STAD. The variations in PTTG mRNA expression throughout STAD tumor stages are shown using violin plots. One-way analysis of variance was used to test for statistical significance (ANOVA). It was determined that a *p* value of 0.01 was statistically significant. (b) Staging of STAD according to PTTG mRNA expression and clinicopathological stages (UALCAN). (c) Nodal metastases and PTTG mRNA expression in patients with STAD (UALCAN). ^∗^*p* < 0.05 and ^∗∗∗^*p* < 0.001; NS: no sense.

**Figure 4:** mRNA expression of PTTGs in GC patients has prognostic value (Kaplan-Meier plotter). The survival curves of GC patients were plotted in three different ways: for overall survival, progression-free survival, and survival after disease progression. JetSet's top-tier probe set was selected for this investigation. The optimal cutoff for dividing patients was determined by an algorithm. The OS curve was labeled as “high” if the expression level was above the cutoff value and as “low” if the expression level was below the cutoff value. Significant results were considered to be at the *p* < 0.05 level. Postprogression survival (PPS) is the time between the occurrence of the first symptom and the patient's death.

**Figure 5:** Overall survival (OS), disease-free survival (DFS), progression-free survival (PFS), and disease-specific survival (DSS) of individuals with STAD, as affected by PTTG gene mutations (cBioPortal). (a) Here is a rundown of the many forms of cancer associated with PTTG mutations. Gene changes in PTTGs were found in 24.64 percent of 69 instances with tubular STAD. Mutations in green, gene amplifications in red, profound deletions in blue, elevated levels of mRNA in pink, and numerous changes in grey. (b) Research into PTTG gene mutations in GC. Out of 412 STAD patients studied, 16 percent had inherited mutations in their STAT3 gene. Mutation rates for PTTG1, PTTG2, and PTTG3p were 6%, 5%, and 9%, respectively. Punctuation mutations are grey while missense mutations are green. Gene duplications are shown in green and large deletions in blue. (c–f) Survival, progression, and death rates were analyzed using Kaplan-Meier plots separated by the presence or absence of mutations in the PTTG gene.

**Figure 6:** Immune infiltrates are linked to PTTG expression in gastric cancer (TIMER). (a–c) Immune cell infiltration is associated with the expression of PTTGs (PTTG1, PTTG2, and PTTG3P) in patients with STAD. Pearson's correlation was used for the analysis of the correlation. Immune cell infiltration's prognostic relevance in gastric cancer (d).

**Figure 7:** Family member interactions within the PTTG family tree. (a) Gene-gene interaction network of individual PTTGs (GeneMANIA). (b) The PTTG protein-protein interaction network.

**Figure 8:** Patients with STAD: a functional enrichment analysis of PTTGs (DAVID). Top 10 GO term enrichment study findings as a bubble graphic, broken down into biological process (a), cellular component (b), and molecular function (c). (d) Pie chart displaying the top 10 enriched KEGG pathways. Name of a GO term function or KEGG pathway (*y*-axis); quantity of genes in the network that have been assigned to that word as a proportion of the total number of genes; genes with a corresponding GO term function or KEGG pathway are the “bubble size.” Important metabolic pathways were gleaned from gene counts and *p* values.

**Table 1:** Gastric cancer and healthy gastric tissues exhibit striking differences in the transcription level of the PTTG family (Oncomine).

	Type of gastric cancer vs. gastric	Fold change	*p* value	*t*-test	References
PTTG1	Gastric mixed adenocarcinoma vs. normal	2.000	6.17*e* − 07	7.415	Chen et al. [23]
	Gastric mixed adenocarcinoma vs. normal	2.064	0.001	3.433	Cho et al. [24]
	Gastric intestinal-type adenocarcinoma vs. normal	2.321	2.41*e* − 17	11.196	Chen et al. [23]
	Gastric intestinal-type adenocarcinoma vs. normal	1.790	0.002	3.125	Cho et al. [24]
	Gastric intestinal-type adenocarcinoma vs. normal	2.631	2.24*e* − 10	7.587	D'Errico et al. [25]
	Diffuse gastric adenocarcinoma vs. normal	2.367	1.98*e* − 06	5.426	Cho et al. [24]
PTTG2	Gastric cancer vs. normal	1.706	0.002	2.986	Cui et al. (2011)
PTTG3P	Diffuse gastric adenocarcinoma vs. normal	2.323	3.67*e* − 05	4.615	Cho et al. [24]

**Table 2:** Evaluation of the association between PTTG expression and clinical prognosis in gastric cancer using the Kaplan-Meier plotting method and other clinicopathological variables.

Clinicopathological characteristics	PTTG1			PTTG2		PTTG3P	
	*N*	Overall survival (*n* = 881)					
		Hazard ratio	*p* value	Hazard ratio	*p* value	Hazard ratio	*p* value
Sex							
Female	244	0.44 (0.29-0.65)	3.70*E* − 05	1.64 (1.16-2.33)	0.0049	0.56 (0.39-0.81)	0.0019
Male	566	0.79 (0.64-0.98)	0.032	1.43 (1.15-1.77)	0.001	0.67 (0.53-0.85)	8.00*E* − 04
Stage							
1	69	0.22 (0.05-0.97)	0.028	3.5 (0.99-12.34)	0.038	0.34 (0.12-0.92)	0.027
2	145	0.53 (0.28-0.98)	0.039	1.6 (0.89-2.9)	0.12	0.43 (0.23-0.78)	0.0044
3	319	0.6 (0.45-0.8)	0.00051	1.4 (1.04-1.86)	0.023	0.68 (0.51-0.9)	0.0075
4	152	0.54 (0.35-0.82)	0.0034	0.75 (0.51-1.11)	0.15	0.64 (0.42-0.98)	0.037
Stage T							
2	253	0.61 (0.4-0.93)	0.021	1.43 (0.86-2.39)	0.16	0.52 (0.34-0.8)	0.0022
3	208	0.69 (0.47-0.99)	0.044	1.15 (0.82-1.62)	0.42	0.68 (0.49-0.96)	0.029
4	39	0.44 (1.09-1.03)	0.054	0.7 (0.28-1.79)	0.46	0.63 (0.27-1.49)	0.29
Stage N							
0	76	0.25 (0.07-0.84)	0.015	3.87 (1.65-9.08)	0.00083	0.46 (0.2-1.08)	0.068
1	232	0.5 (0.33-0.75)	0.00072	1.45 (0.96-2.18)	0.076	0.46 (0.31-0.7)	0.00021
2	129	0.59 (0.37-0.93)	0.021	0.54 (0.33-0.87)	0.11	1.46 (0.85-2.58)	0.16
3	76	0.49 (0.29-0.85)	0.0094	0.58 (0.32-1.06)	0.071	0.48 (0.27-0.87)	0.013
1 + 2 + 3	437	0.58 (0.45-0.76)	4.50*E* − 05	1.14 (0.88-1.48)	0.33	0.55 (0.42-0.73)	1.20*E* − 05
Stage M							
0	459	0.55 (0.41-0.73)	4.30*E* − 05	1.31 (1-1.73)	0.053	0.53 (0.4-0.7)	5.60*E* − 06
1	58	0.53 (0.29-0.98)	0.039	0.7 (0.37-1.32)	0.26	0.52 (0.27-1)	0.045
Lauren classification							
Intestinal	336	0.55 (0.4-0.76)	0.00024	1.61 (1.17-2.22)	0.0031	0.5 (0.36-0.68)	9.90*E* − 06
Diffuse	248	0.63 (0.44-0.9)	0.01	1.33 (0.95-1.88)	0.098	0.6 (0.4-0.89)	0.01
Differentiation							
Poor	166	1.75 (1.17-2.63)	0.0057	1.28 (0.85-1.92)	0.23	1.2 (0.8-1.81)	0.37
Moderate	67	0.63 (0.31-1.25)	0.18	0.63 (0.33-1.2)	0.15	0.51 (0.26-0.99)	0.042
High	32	0.57 (0.23-1.43)	0.23	1.55 (0.65-3.69)	0.32	0.31 (0.12-0.8)	0.011
Treatment							
Surgery alone	393	0.6 (0.44-0.81)	7.00*E* − 04	1.2 (0.9-1.6)	0.21	0.61 (0.46-0.82)	0.00072
5 FU-based adjuvant	157	2.12 (1.4-3.21)	0.00032	1.56 (1.1-2.21)	0.011	1.87 (1.26-2.77)	0.0016
Other adjuvant	80	0.49 (0.2-1.18)	0.11	2.84 (1.09-7.41)	0.025	0.29 (0.07-1.25)	0.076
HER2 status							
Positive	424	0.75 (0.56-1.01)	0.053	1.41 (1.06-1.88)	0.016	0.75 (0.57-1)	0.05
Negative	641	0.64 (0.51-0.81)	0.00012	1.59 (1.25-2.01)	0.00011	0.62 (0.49-0.78)	2.70*E* − 05

**Table 3:** Correlation analysis between PTTGs and biomarkers of immune cells in TIMER.

Description	Gene markers	PTTG1				PTTG2				PTTG3P			
		None		Purity		None		Purity		None		Purity	
		Cor	*p*	Cor	*p*	Cor	*p*	Cor	*p*	Cor	*p*	Cor	*p*
CD8+T cell	CD8A	-0.036	4.65*E* − 01	-0.034	5.11*E* − 01	0.131	∗	0.125	1.50*E* − 02	-0.016	7.53*E* − 01	-0.022	6.73*E* − 01
	CD8B	0.019	6.94*E* − 01	0.031	5.54*E* − 01	0.107	2.90*E* − 02	0.111	3.01*E* − 02	0.026	5.96*E* − 01	0.021	6.78*E* − 01
T cell (general)	CD3D	-0.017	7.24*E* − 01	0.002	9.74*E* − 01	0.210	∗∗∗	0.211	∗∗∗	0.086	8.07*E* − 02	0.098	5.72*E* − 02
	CD3E	-0.080	1.05*E* − 01	-0.065	2.06*E* − 01	0.145	∗	0.138	∗	-0.036	4.71*E* − 01	-0.032	5.32*E* − 01
	CD2	-0.050	3.06*E* − 01	-0.042	4.12*E* − 01	0.213	∗∗∗	0.209	∗∗∗	0.091	6.34*E* − 02	0.101	5.02*E* − 02
B cell	CD19	-0.187	^∗∗^	-0.185	∗∗	0.125	1.11*E* − 02	0.097	5.97*E* − 02	-0.034	4.90*E* − 01	-0.035	4.95*E* − 01
	CD79A	-0.216	^∗∗∗^	-0.215	∗∗∗	0.109	2.65*E* − 02	0.087	8.97*E* − 02	-0.037	4.47*E* − 01	-0.034	5.15*E* − 01
Monocyte	CD86	-0.036	4.68*E* − 01	-0.027	5.95*E* − 01	0.216	∗∗∗	0.224	∗∗∗	0.173	∗∗	0.188	∗∗
	CD115(CSF1R)	-0.245	^∗∗∗^	-0.251	∗∗∗	0.156	∗	0.152	∗	0.029	5.53*E* − 01	0.034	5.04*E* − 01
TAM	CCL2	-0.174	^∗∗^	-0.175	∗∗	0.103	3.66*E* − 02	0.110	3.21*E* − 02	-0.017	7.26*E* − 01	-0.012	8.23*E* − 01
	CD68	-0.093	5.90*E* − 02	-0.095	6.37*E* − 02	-0.013	7.89*E* − 01	-0.034	5.11*E* − 01	0.029	5.50*E* − 01	0.033	5.20*E* − 01
	IL10	-0.095	5.20*E* − 02	-0.085	9.84*E* − 02	0.172	∗∗	0.169	∗∗	0.113	2.19*E* − 02	0.104	4.38*E* − 02
M1 macrophage	INOS (NOS2)	0.128	^∗^	0.122	1.79*E* − 02	-0.005	9.15*E* − 01	-0.003	9.55*E* − 01	0.057	2.50*E* − 01	0.036	4.86*E* − 01
	IRF5	-0.159	^∗^	-0.162	∗	-0.009	8.57*E* − 01	-0.020	6.92*E* − 01	-0.069	1.59*E* − 01	-0.072	1.61*E* − 01
	COX2 (PTGS2)	-0.068	1.69*E* − 01	-0.066	1.99*E* − 01	0.102	3.71*E* − 02	0.114	2.67*E* − 02	0.093	5.92*E* − 02	0.111	3.11*E* − 02
M2 macrophage	CD163	-0.134	^∗^	-0.137	∗	0.201	∗∗∗	0.206	∗∗∗	0.108	2.72*E* − 02	0.125	1.51*E* − 02
	VSIG4	-0.130	^∗^	-0.140	∗	0.174	∗∗	0.179	∗∗	0.103	3.58*E* − 02	0.111	3.01*E* − 02
	MS4A4A	-0.182	^∗∗^	-0.179	∗∗	0.227	∗∗∗	0.229	∗∗∗	0.140	∗	0.148	∗
Neutrophils	CD66b (CEACAM8)	0.056	2.58*E* − 01	0.057	2.70*E* − 01	0.189	∗∗	0.199	∗∗∗	0.280	∗∗∗	0.256	∗∗∗
	CD11b (ITGAM)	-0.217	^∗∗∗^	-0.214	∗∗∗	0.143	∗	0.142	∗	0.028	5.76*E* − 01	0.039	4.54*E* − 01
	CCR7	-0.278	^∗∗∗^	-0.273	∗∗∗	0.181	∗∗	0.180	∗∗	-0.005	9.13*E* − 01	-0.004	9.34*E* − 01
Natural killer cell	KIR2DL1	0.066	1.79*E* − 01	0.074	1.48*E* − 01	0.209	∗∗∗	0.219	∗∗∗	0.223	∗∗∗	0.201	∗∗∗
	KIR2DL3	0.047	3.38*E* − 01	0.054	2.97*E* − 01	0.296	∗∗∗	0.302	∗∗∗	0.323	∗∗∗	0.301	∗∗∗
	KIR2DL4	0.250	^∗∗∗^	0.269	∗∗∗	0.148	∗	0.140	∗	0.178	∗∗	0.177	∗∗
	KIR3DL1	0.013	7.89*E* − 01	-0.007	8.89*E* − 01	0.159	∗	0.160	∗	0.138	∗	0.137	∗
	KIR3DL2	0.048	3.33*E* − 01	0.038	4.64*E* − 01	0.260	∗∗∗	0.264	∗∗∗	0.194	∗∗∗	0.173	∗∗
	KIR3DL3	0.114	1.98*E* − 02	0.116	2.36*E* − 02	0.082	9.49*E* − 02	0.070	1.71*E* − 01	0.171	∗∗	0.115	2.54*E* − 02
	KIR2DS4	0.086	8.05*E* − 02	0.096	6.09*E* − 02	0.189	∗∗	0.183	∗∗	0.166	∗∗	0.169	∗∗
Dendritic cell	HLA-DPB1	-0.125	1.07*E* − 02	-0.113	2.85*E* − 02	0.168	∗∗	0.165	∗	0.019	6.98*E* − 01	0.025	6.27*E* − 01
	HLA-DQB1	-0.035	4.77*E* − 01	-0.018	7.20*E* − 01	0.072	1.43*E* − 01	0.061	2.35*E* − 01	0.006	9.06*E* − 01	0.008	8.82*E* − 01
	HLA-DRA	-0.034	4.84*E* − 01	-0.017	7.35*E* − 01	0.187	∗∗	0.182	∗∗	0.079	1.06*E* − 01	0.090	7.98*E* − 02
	HLA-DPA1	-0.074	1.33*E* − 01	-0.060	2.43*E* − 01	0.166	∗∗	0.160	∗	0.052	2.90*E* − 01	0.057	2.70*E* − 01
	BCDA-1 (CD1C)	-0.394	^∗∗∗^	-0.403	∗∗∗	0.185	∗∗	0.176	∗∗	0.000	9.92*E* − 01	0.000	9.98*E* − 01
	BDCA-4 (NRP1)	-0.296	^∗∗∗^	-0.291	∗∗∗	0.193	∗∗∗	0.205	∗∗∗	0.015	7.64*E* − 01	0.029	5.72*E* − 01
	CD11c (ITGAX)	-0.140	^∗^	-0.125	1.45*E* − 02	0.182	∗∗	0.181	∗∗	0.117	1.73*E* − 02	0.122	1.74*E* − 02
Th1	T-bet (TBX21)	-0.033	5.08*E* − 01	-0.034	5.08*E* − 01	0.136	∗	0.121	1.89*E* − 02	0.026	6.01*E* − 01	0.013	8.06*E* − 01
	STAT4	-0.172	^∗∗^	-0.165	∗	0.286	∗∗∗	0.300	∗∗∗	0.134	∗	0.142	∗
	STAT1	0.245	^∗∗∗^	0.244	∗∗∗	0.133	∗	0.121	1.88*E* − 02	0.127	∗	0.118	2.20*E* − 02
	IFN-*γ* (IFNG)	0.273	^∗∗∗^	0.281	∗∗∗	0.171	∗∗	0.160	∗	0.174	∗∗	0.179	∗∗
	TNF-*α* (TNF)	0.026	5.92*E* − 01	0.036	4.90*E* − 01	0.006	8.96*E* − 01	-0.017	7.43*E* − 01	0.026	5.93*E* − 01	0.039	4.50*E* − 01
Th2	GATA3	-0.171	^∗∗^	-0.160	∗	0.180	∗∗	0.188	∗∗	-0.004	9.35*E* − 01	-0.007	8.93*E* − 01
	STAT6	-0.206	^∗∗∗^	-0.213	∗∗∗	0.014	7.78*E* − 01	0.012	8.21*E* − 01	-0.140	∗	-0.139	∗
	STAT5A	-0.201	^∗∗∗^	-0.205	∗∗∗	0.170	∗∗	0.154	∗	-0.042	3.94*E* − 01	-0.042	4.12*E* − 01
	IL13	-0.003	9.57*E* − 01	-0.005	9.25*E* − 01	0.031	5.26*E* − 01	0.019	7.10*E* − 01	-0.041	4.04*E* − 01	-0.053	3.02*E* − 01
Tfh	BCL6	-0.371	^∗∗∗^	-0.370	∗∗∗	0.157	∗	0.163	∗	-0.027	5.84*E* − 01	-0.012	8.19*E* − 01
	IL21	0.121	1.35*E* − 02	0.142	∗	0.193	∗∗∗	0.174	∗∗	0.160	∗	0.172	∗∗
Th17	STAT3	-0.231	^∗∗∗^	-0.237	∗∗∗	0.114	1.99*E* − 02	0.104	4.22*E* − 02	-0.040	4.14*E* − 01	-0.035	4.97*E* − 01
	IL17A	0.171	^∗∗^	0.175	∗∗	-0.085	8.40*E* − 02	-0.112	2.90*E* − 02	0.051	3.01*E* − 01	0.056	2.73*E* − 01
Treg	FOXP3	0.012	8.00*E* − 01	0.022	6.74*E* − 01	0.035	4.75*E* − 01	0.017	7.36*E* − 01	-0.035	4.72*E* − 01	-0.047	3.61*E* − 01
	CCR8	-0.077	1.16*E* − 01	-0.080	1.20*E* − 01	0.182	∗∗	0.176	∗∗	0.124	1.14*E* − 02	0.125	1.51*E* − 02
	STAT5B	-0.362	^∗∗∗^	-0.364	∗∗∗	0.156	∗	0.159	∗	-0.072	1.43*E* − 01	-0.072	1.64*E* − 01
	TGF*β* (TGFB1)	-0.206	^∗∗∗^	-0.192	^∗∗^	0.042	3.96*E* − 01	0.042	4.12*E* − 01	-0.106	3.16*E* − 02	-0.104	4.22*E* − 02
T cell exhaustion	PD-1 (PDCD1)	0.061	2.17*E* − 01	0.072	1.63*E* − 01	0.058	2.39*E* − 01	0.042	4.19*E* − 01	-0.057	2.46*E* − 01	-0.069	1.82*E* − 01
	CTLA4	0.110	2.57*E* − 02	0.124	1.61*E* − 02	0.184	∗∗	0.177	∗∗	0.138	∗	0.147	∗
	LAG3	0.146	^∗^	0.152	^∗^	0.095	5.27*E* − 02	0.081	1.15*E* − 01	0.013	7.94*E* − 01	-0.001	9.82*E* − 01
	TIM-3 (HAVCR2)	-0.004	9.35*E* − 01	0.004	9.37*E* − 01	0.182	∗∗	0.181	∗∗	0.157	∗	0.158	∗
	GZMB	0.305	^∗∗∗^	0.322	^∗∗∗^	0.121	1.39*E* − 02	0.105	4.05*E* − 02	0.146	∗	0.147	∗

TAM: tumor-associated macrophage; Th: T helper cell; Tfh: follicular helper T cell; Treg: regulatory T cell. *R* value of Spearman's correlation coefficient; correlation with no modification; correlation after using the purity criterion. ^∗^*p* < 0.01; ^∗∗^*p* < 0.001; ^∗∗∗^*p* < 0.0001.

## Data Availability

The datasets used and/or analyzed during the current study are available from the corresponding author on reasonable request.
